# Comparing the Prognostic Value of Stress Myocardial Perfusion Imaging by Conventional and Cadmium-Zinc Telluride Single-Photon Emission Computed Tomography through a Machine Learning Approach

**DOI:** 10.1155/2021/5288844

**Published:** 2021-10-16

**Authors:** Valeria Cantoni, Roberta Green, Carlo Ricciardi, Roberta Assante, Leandro Donisi, Emilia Zampella, Giuseppe Cesarelli, Carmela Nappi, Vincenzo Sannino, Valeria Gaudieri, Teresa Mannarino, Andrea Genova, Giovanni De Simini, Alessia Giordano, Adriana D'Antonio, Wanda Acampa, Mario Petretta, Alberto Cuocolo

**Affiliations:** ^1^Department of Advanced Biomedical Sciences, University of Naples Federico II, Naples, Italy; ^2^Department of Electrical Engineering and Information Technology, University of Naples Federico II, Naples, Italy; ^3^Bioengineering Unit, Institute of Care and Scientific Research Maugeri, Telese Terme, Campania, Italy; ^4^Department of Chemical, Materials and Production Engineering, University of Naples Federico II, Naples, Italy; ^5^Institute of Biostructure and Bioimaging, National Council of Research, Naples, Italy; ^6^IRCCS SDN, Naples, Italy

## Abstract

We compared the prognostic value of myocardial perfusion imaging (MPI) by conventional- (C-) single-photon emission computed tomography (SPECT) and cadmium-zinc-telluride- (CZT-) SPECT in a cohort of patients with suspected or known coronary artery disease (CAD) using machine learning (ML) algorithms. A total of 453 consecutive patients underwent stress MPI by both C-SPECT and CZT-SPECT. The outcome was a composite end point of all-cause death, cardiac death, nonfatal myocardial infarction, or coronary revascularization procedures whichever occurred first. ML analysis performed through the implementation of random forest (RF) and *k*-nearest neighbors (KNN) algorithms proved that CZT-SPECT has greater accuracy than C-SPECT in detecting CAD. For both algorithms, the sensitivity of CZT-SPECT (96% for RF and 60% for KNN) was greater than that of C-SPECT (88% for RF and 53% for KNN). A preliminary univariate analysis was performed through Mann-Whitney tests separately on the features of each camera in order to understand which ones could distinguish patients who will experience an adverse event from those who will not. Then, a machine learning analysis was performed by using Matlab (v. 2019b). Tree, KNN, support vector machine (SVM), Naïve Bayes, and RF were implemented twice: first, the analysis was performed on the as-is dataset; then, since the dataset was imbalanced (patients experiencing an adverse event were lower than the others), the analysis was performed again after balancing the classes through the Synthetic Minority Oversampling Technique. According to KNN and SVM with and without balancing the classes, the accuracy (*p* value = 0.02 and *p* value = 0.01) and recall (*p* value = 0.001 and *p* value = 0.03) of the CZT-SPECT were greater than those obtained by C-SPECT in a statistically significant way. ML approach showed that although the prognostic value of stress MPI by C-SPECT and CZT-SPECT is comparable, CZT-SPECT seems to have higher accuracy and recall.

## 1. Introduction

Risk stratification by noninvasive cardiac imaging has become increasingly important to optimize management and outcome in patients with coronary artery disease (CAD) [1]. Previous research indicated that stress single-photon emission computed tomography (SPECT) myocardial perfusion imaging (MPI) has been the most widely used nuclear cardiac imaging technique for the noninvasive assessment of cardiac disease, including the prognosis and choice of the most appropriate treatment strategies for patients with CAD [2]. Conventional- (C-) SPECT systems utilize sodium iodide crystals and parallel-hole collimators. This approach presents some technical limits; for instance, we can mention extended imaging time, low spatial resolution, and large doses of radiopharmaceuticals [3]. Recently, these limitations have been overcome with the introduction of gamma cameras with semiconductor cadmium-zinc-telluride (CZT) allowed to directly convert radiation into electric signals, bringing an improvement in image accuracy and acquisition time [4, 5].

Previous studies showed that CZT-SPECT findings can be used for risk stratification of patients referred to MPI for suspected or known CAD. Lima et al. [6] demonstrated that CZT-SPECT and C-SPECT provide similar prognostic results, with lower prevalence of hard events in patients with normal scan [6]. Yokota et al. [7] showed that the prognostic value of normal stress-only CZT-SPECT is at least comparable and may be even better than that of normal C-SPECT [7].

These biomedical technologies can produce big amount of data and, nowadays, different techniques have been used to obtain as much information as possible from data and signals [8–12]. Introducing machine learning (ML) in the healthcare sector can help clinicians in diagnosis and therapy planning, as well as in management of resources [13, 14]. Several studies have been conducted to test CAD detection using ML algorithms and to predict patient outcome [15–18]. An innovative approach is to use ML models to compare the performance of biomedical technologies, and an evaluation of the performance in terms of diagnostic power has already been reported [19, 20], demonstrating CZT-SPECT has a better ability to detect CAD. To the best of our knowledge, the prognostic value of CZT-SPECT and C-SPECT has not been investigated to date by using ML techniques.

Therefore, the purposes of the present investigation were as follows:

1. To evaluate the prognostic value of C-SPECT and CZT-SPECT using ML-based approaches in patients with suspected or known CAD
2. To compare the prognostic performance of these biomedical instrumentations through ML

This use of ML—in this particular case, aimed at compering two biomedical technologies—represents, to authors' best knowledge, one of the first attempts in literature.

## 2. Materials and Methods

### 2.1. Patients

Between February 2016 and May 2017, a total of 453 consecutive patients with suspected or known CAD were submitted by referring physicians to stress MPI for assessment of myocardial ischemia. For overall population, clinical history and cardiac risk factors were collected. Patients with a previous history of myocardial infarction, revascularization procedures, or a diagnosed atherosclerotic coronary disease were considered to have known CAD. The review committee of our institution approved the study (Protocol Number 110/17), and all patients gave informed consent.

### 2.2. Study Protocol

All patients were submitted to stress technetium-99m sestamibi-gated SPECT MPI by physical exercise or dipyridamole stress test, according to the recommendations of the European Association of Nuclear Medicine and European Society of Cardiology [21]. The protocol followed in this paper was the same employed in our previous research [20]. All patients underwent MPI by both C-SPECT and CZT-SPECT systems according to a randomized scheme in 1 : 1 ratio that determined which camera was used for first acquisition. For C-SPECT, a dual-head rotating gamma camera (E.CAM, Siemens Medical Systems, Hoffman Estates, IL, USA) was used. The acquisition time was 20 min for both stress and rest images. For CZT-SPECT (D-SPECT, Spectrum Dynamics, Caesarea, Israel), recordings were obtained using 9 pixilated CZT crystal detector columns mounted vertically spanning a 90 geometry. Scan duration was lower than 10 minutes for stress and lower than 5 minutes for rest imaging.

An automated software program (e-soft, 2.5, QGS/QPS, Cedars- Sinai Medical Center, Los Angeles, CA) was utilized to compute left ventricular (LV) volumes and ejection fraction (EF) and the scores incorporating both the extent and severity of perfusion defects, employing a standard segmentation of the 17 myocardial regions. The extent and grade of the quantitative defect were determined based on sex-specific normal limits while adding the scores of the 17 segments (from 0 for normal to 4 for absent perfusion) of the stress images allowed us to compute the summed stress score (SSS). A poststress LVEF greater than 45% and a SSS lower than 3 were considered normal.

### 2.3. Follow-Up Data

A follow-up questionnaire was collected by calling all patients by examinators blinded to patient's test results. The outcomes evaluated as endpoints were all-cause death, cardiac death, nonfatal myocardial infarction, or coronary revascularization procedures whichever occurred first. Cardiac death occurred subsequently to acute myocardial infarction, congestive heart failure, and cardiac interventional procedure related. Myocardial infarction was recorded when chest pain or equivalent symptom complex, positive cardiac biomarkers, or typical electrocardiographic changes were reported [22]. The length of follow-up was determined according to the date of the last medical visit.

### 2.4. Statistical Analysis

Statistical analyses were performed by using IBM SPSS statistics software (v. 26), both to test data distribution and to perform statistical tests. The process was carried out separately on both the parameters of the C-SPECT and the CZT-SPECT. First, the Kolmogorov-Smirnov test was performed to test data normality, in order to understand the type of test to be used (parametric or nonparametric): in particular, normality was tested for all parameters, for both groups, and for both camera types. Subsequently, a two-tailed *t*-test was performed for parameters with a normal distribution, while Mann-Whitney test was performed for the remaining parameters, and both tests were conducted considering a significance level of 0.05. After the use of ML algorithms, a chi-square test was used in order to compare the performances of different the models, trained with C-SPECT and the CZT-SPECT data, and to understand if there were statistical differences among them. The results are shown and discussed in the “Results” and “Discussion” sections, respectively.

### 2.5. Machine Learning Algorithms

The ML analysis was performed by using the Classification Learning App, provided by Matlab (v. 2019b), which trains models to classify data using supervised ML. The 10-fold crossvalidation was used to train and test the models; the dataset was divided into 10 groups of data, 9 were used for training the model and one group for testing it; the procedure was repeated 10 times, and the evaluation metrics are computed by averaging all those obtained [23]. The tree-based approach has shown in literature great results not only in the cardiologic context in cases such as diagnosis [24–26], prognosis [27, 28], and comparison of biomedical technologies [19, 20] but also in other medical specialties [29–31]. The classification tree is a simple and effective model consisting of nodes, branches, and leaves: each node has a rule that the data is routed along several branches while the leaves represent the output of the system [32].

Random forests (RF) model is part of the ensemble algorithms and allows to train together a set number of decision trees using the technique of Bootstrap Aggregation; this model turns out to have better accuracy than the single weak learner and reduces the chance of overfitting [33]. *K*-nearest neighbor (KNN) algorithm is a distance-based method. In fact, an example's membership in a class is determined by proximity to other known class examples. The critical aspect is the choice of the value of *k* that is the number of neighbors to consider for the decision [34]. Support vector machine (SVM) is a classification model that is based on finding the best surface that allows you to separate the two classes. In particular, the algorithm tries to maximize the margin between classes, the space that separates them, and in this way, bases learning on the most difficult examples, decreasing the influence of outliers [35]. Naïve Bayes (NB) was also employed in this study; it is a well-known algorithm based on the a priori probability theorem [36], thus being a completely different algorithm compared to the previous ones. These algorithms were used to predict an adverse event by using the features of the two cameras, and then, the evaluation metrics were compared through a statistical test for proportions in order to understand which one had the best capacity to detect the adverse event.

The present dataset is unbalanced; indeed, people with adverse events turned out to be much less than those with no events. In the literature, the problems that arise in training ML models using unbalanced data are well known [37, 38]. To deal with this problem, the Synthetic Minority Oversampling Technique (SMOTE) [39] was used; this oversampling technique generates new artificial data of the minority class, on the basis of those already present, allowing to rebalance the dataset. After that, the training phase of the models was repeated. This can be considered fair because it will be employed on both cameras allowing a fair comparison; moreover, the aim of the study is to compare C-SPECT and the CZT-SPECT rather than build the best prognostic model.

To evaluate the performance of the models, several metrics [40] were used: accuracy, sensitivity or recall, specificity, and precision. Furthermore, area under the curve (AUC) receiver-operating characteristic (ROC) was computed because it is a good method to assess model performance [41]. In addition, a feature selection process was performed to understand which parameters resulted more significant in reference to the target variable. We tested 14 features: perfusion parameters as SSS, summed rest score (SRS), summed difference score (SDS), and total perfusion defect (TPD) and functional parameters as systolic wall motion (SWM), systolic wall thickening (SWT), end-diastolic volume (EDV), end-systolic volume (ESV), and EF. In particular, two algorithms were used: Maximum Relevance–Minimum Redundancy (MRMR) that selects the variables with the most relevance to the destination one by calculating the mutual information of the parameters [42] and chi-square independence test [43].

## 3. Results

### 3.1. Patient Characteristics and Outcome

The clinical characteristics of patient population are shown in Table 1. The study group comprised 204 (45%) patients with suspected CAD and 249 (55%) with known CAD. The mean follow-up was 2.5 ± 0.5 years. During follow-up, 41 events occurred. The events were cardiac death in 1 patient, nonfatal myocardial infarction in 5, coronary revascularization procedures in 20, and 15 all-cause of death.

### 3.2. Statistical Analysis

The first step was to evaluate the possible normal distribution of the features between patients with events and patients with no events evaluated by both cameras, applying Kolmogorov-Smirnov test. The test revealed that, among the features of C-SPECT, only stress and rest EF (*p* value > 0.05) showed a normal distribution for both groups; similarly, no features of CZT-SPECT resulted to have a Gaussian distribution. Therefore, *t*-test was used only for stress and rest EF by C-SPECT, while Mann-Whitney test was performed for all other parameters, and the results are reported in Table 2.

### 3.3. Machine Learning Analysis

The ML analysis was conducted separately and by using a 10-fold crossvalidation for C-SPECT and CZT-SPECT, both before and after SMOTE application in order to compare camera's performance with and without the augmentation of the dataset. The evaluation metrics regarding the models without SMOTE are reported in Table 3. Among the ML algorithms used for the analysis, RF reached the highest value of accuracy (90.3% and 90.1%, respectively, for C-SPECT and CZT-SPECT) and recall (98.5% and 99.0%, respectively, for C-SPECT and CZT-SPECT), but it presented the lowest value of specificity (7.3% and 0%, respectively, for C-SPECT and CZT-SPECT), showing a low capacity to detect adverse future events. Despite achieving these performances, statistically significant differences between the two cameras were not available, and this was also verified for Tree, SVM, and NB models. KNN model had an accuracy and recall lower than RF for both cameras (accuracy of 74.4% and 80.8%, recall of 78.6% and 87.4%, respectively, for C-SPECT and CZT-SPECT) but higher specificity (ranging from 14.6%, in CZT-SPECT, to 31.7% in C-SPECT). Nevertheless, the accuracy and the capacity to detect the absence of adverse event were statistically significant in favour of the CZT camera (*p* value = 0.021 for accuracy and *p* value = 0.001 for recall). These results were influenced by the imbalanced nature of the datasets; indeed, although accuracy and recall were high, they were affected by the bias introduced by the presence of a majority class for subjects with a negative prognosis, as also validated by the low AUCROC values of the models (ranging from 0.53 to 0.60 for C-SPECT and from 0.50 to 0.61 for CZT-SPECT). To overcome this issue, the dataset was balanced by introducing artificial samples of the minority class (patients with future adverse events), generated with SMOTE. The evaluation metrics values are reported in Table 4. The overall performance of classifiers increased significantly with a balanced dataset, especially in terms of specificity and AUCROC. Considering the C-SPECT, RF reached the highest values of accuracy (93.4%), recall (90.3%), and AUCROC (0.99), while SVM and KNN reached higher values of specificity (95.0% and 99.8%, respectively). Regarding CZT camera models performances, SVM classifier reached the highest values of accuracy (94.5%), recall (92.2%), and specificity (96.8%). Moreover, SVM turned out to have statistically significant performances: the accuracy and the recall showed a statistical significance in favor of the CZT-camera (*p* value = 0.016 for accuracy and *p* value = 0.028 for recall), while, despite showing in CZT-SPECT a higher capacity to detect adverse events, the specificity of SVM was not found to be statistically significant (*p* value = 0.279).

## 4. Discussion

To our knowledge, this is the first study using ML approach to compare the prognostic value of two technologies used in clinical routine practice (C-SPECT and CZT-SPECT) in patients with suspected or known CAD. Indeed, the ML analysis did not aim to create the best model to predict adverse events because, probably, it would not have been possible considering the highly unbalanced nature of the dataset. The aim was to test the feasibility of the cameras in predicting adverse future events in order to understand which could be the one with the better performance.

Although a similar evaluation has already been performed, ML techniques have never been used. Lima et al. [6] compared the prognostic value of MPI using an ultrafast protocol with low radiation in CZT-SPECT and a C-SPECT in different groups of patients. They concluded that the new protocol of MPI in CZT-SPECT showed similar prognostic results to those obtained in dedicated cardiac Na-I SPECT camera, with lower prevalence of hard events in patients with normal scan. Similarly, Yokota et al. [7] compared the prognosis of patients with normal stress-only at both CZT-SPECT and C-SPECT. They showed that the prognostic value of normal stress-only CZT-SPECT is at least comparable and may be even better than that of normal stress-only C-SPECT. In a recent study, Liu et al. [44] showed that ultralow dose thallium perfusion imaging using CZT-SPECT provides good prognostic results, with a more severe prognosis in patients with abnormal MPI.

However, ML has been recently employed for the comparison of biomedical technologies. In previous studies using ML techniques to compare the diagnostic performance of C-SPECT and CZT-SPECT, we highlighted how algorithms trained with CZT-SPECT data achieved better accuracy, recall, and specificity than C-SPECT [19, 20]. Concerning the ML models, it has been observed that they generally present a high accuracy and recall. In particular, accuracy (*p* value = 0.021) and recall (*p* value = 0.001) were statistically significant for CZT-SPECT through the KNN algorithm. This result would demonstrate that CZT-SPECT has better performance to detect the absence of adverse event. To enhance the results obtained on the unbalanced dataset, a process of rebalancing the dataset was applied using SMOTE and repeating all the ML analyses. As expected, the performance of all models improved significantly for both cameras after rebalancing. However, SVM showed marked differences in all metrics values: accuracy, recall, and specificity had higher values in CZT-SPECT than C-SPECT. In particular, accuracy and recall were statistically significant in favour of CZT-SPECT (accuracy *p* value = 0.016, recall *p* value = 0.028). Therefore, even considering the balanced data, CZT-SPECT proved to achieve a better accuracy and ability in predicting the absence of adverse event. It is likely that patients affected by an adverse event had a particular pattern of input variables which have allowed instance-based algorithms (KNN and SVM) to capture the outcome better than tree-based and probability-based algorithms. As regards the computational costs and the runtime of our models, there was no specific problem because all the models followed a simple workflow without applying heavy preprocessing algorithms (such as backward or forward feature selection methods). Indeed, all the models required less than a minute to be run.

The novel CZT technique provides patients with several advantages, as lower radiation dose and imaging time. Moreover, the higher energy and intrinsic spatial resolution of CZT detectors lead to lower artifacts and need for rest imaging, with a consequent reduction in radiopharmaceutical dosage which enables nuclear MPI to be more cost-effective [45].

### 4.1. Limitations and Future Developments

This study has some limitations that need to be considered. The dataset was strongly imbalanced, to the detriment of patients who present adverse events. It influenced the learning process of the models, introducing biases into evaluation metrics. SMOTE technique has been applied to balance the dataset and overcome these issues. However, the samples introduced were artificial, which represented another limitation. Nevertheless, the aim of the paper was not to evaluate the performance of the models in order to create a tool for clinical support, but to compare the performance of two technologies; therefore, the limitation introduced by the oversampling process is attenuated. Regarding future developments, it would be necessary to try to balance the dataset with original data rather than with artificial samples in order to increase the reliability of the evaluation metrics.

## 5. Conclusions

The novelty introduced in this study was the use of supervised learning techniques to compare the prognostic value of C-SPECT and CZT-SPECT. The results obtained showed that although the prognostic value of the two systems is comparable; CZT-SPECT seems to have higher accuracy and recall.

## Figures and Tables

**Table 1:** Clinical characteristics of patient population.

Characteristic	
Age (years)	64 ± 10
Male gender, *n* (%)	331 (73)
Body mass index ≥ 30 kg/m^2^, *n* (%)	110 (24)
Diabetes, *n* (%)	153 (34)
Dyslipidemia, *n* (%)	333 (74)
Smoking, *n* (%)	196 (43)
Hypertension, *n* (%)	386 (85)
Atypical angina, *n* (%)	162 (36)
Family history of CAD, *n* (%)	231 (51)
Previous myocardial infarction, *n* (%)	148 (33)
Previous revascularization procedures, *n* (%)	173 (38)

Data are presented as mean ± SD or *n* (%) of subjects. CAD: coronary artery disease.

**Table 2:** Univariate statistical analysis of all the parameters of C-SPECT and the CZT-SPECT.

Parameters	C-SPECT			CZT-SPECT		
	Patients with no event	Patients with event	*p* value	Patients with no event	Patients with event	*p* value
SSS	9.90 ± 8.10	15.10 ± 11.50	0.053	9.30 ± 7.70	14.30 ± 11.70	<0.001^∗∗∗^
SRS	6.80 ± 7.90	11.40 ± 11.60	0.163	5.10 ± 7.10	9.30 ± 11.10	0.240
SDS	3.10 ± 3.20	3.00 ± 2.50	0.841	4.10 ± 3.10	4.50 ± 2.80	0.310
TPD	13.10 ± 11.70	20.40 ± 16.70	0.043^∗^	13.10 ± 11.80	20.20 ± 17.30	<0.001^∗∗∗^
Stress SWM	14.90 ± 12.20	18.80 ± 15.00	0.007^∗^	10.70 ± 12.10	14.70 ± 14.10	0.018^∗^
Stress SWT	8.90 ± 9.20	11.70 ± 10.40	0.002^∗^	6.70 ± 8.50	9.10 ± 9.40	0.020^∗^
Stress EDV	92.90 ± 37.80	105.00 ± 51.50	0.031^∗^	106.10 ± 42.40	121.10 ± 57.40	0.044^∗^
Stress ESV	48.10 ± 32.30	60.40 ± 44.80	0.006^∗^	54.70 ± 36.50	71.10 ± 51.50	0.008^∗∗^
Stress EF	52.30 ± 14.20	48.40 ± 15.50	<0.001^∗^	51.30 ± 11.80	46.80 ± 13.10	0.005^∗∗^
Rest SWM	15.40 ± 12.70	21.50 ± 15.00	0.048^∗^	10.20 ± 12.20	15.40 ± 13.00	0.070
Rest SWT	9.40 ± 9.40	12.65 ± 10.30	0.128	6.10 ± 8.30	9.80 ± 13.30	0.110
Rest EDV	91.86 ± 41.05	99.77 ± 41.48	0.493	106.30 ± 45.40	114.10 ± 52.50	0.790
Rest ESV	48.10 ± 35.70	57.60 ± 37.20	0.283	55.30 ± 41.50	65.50 ± 43.90	0.420
Rest EF	51.70 ± 13.80	46.60 ± 14.90	0.098	50.80 ± 12.00	46.90 ± 14.10	0.160

Statistically significant at: ^∗^0.05, ^∗∗^0.001, ^∗∗∗^<0.001. Abbreviations. EDV: end-diastolic volume; EF: ejection fraction; ESV: end-systolic volume; SDS: summed difference score; SRS: summed rest score; SSS: summed stress score; SWM: wall motion; SWT: wall thickening; TPD: total perfusion defect.

**Table 3:** Machine learning analysis and statistical comparison through chi square test for proportions on the original dataset.

		Accuracy (%)	Error (%)	Recall (%)	Specificity (%)
Tree	C-SPECT	87.4	12.6	94.4	17.1
	CZT-SPECT	89.0	11.0	97.1	7.32
	*p* value	0.471		0.057	0.177
KNN	C-SPECT	74.4	25.6	78.6	31.7
	CZT-SPECT	80.8	19.2	87.4	14.6
	*p* value	**0.021**		**0.001**	0.067
SVM	C-SPECT	85.9	14.1	92.2	21.6
	CZT-SPECT	86.5	13.5	92.6	21.6
	*p* value	0.773		0.597	1.000
NB	C-SPECT	83.4	16.6	89.1	26.8
	CZT-SPECT	84.1	15.9	90.1	24.4
	*p* value	0.787		0.649	0.800
RF	C-SPECT	90.3	9.7	98.5	7.3
	CZT-SPECT	90.1	9.9	99.0	0.0
	*p* value	0.591		0.525	0.078

Abbreviations: KNN: *K* nearest neighbor; SVM: support vector machine; NB: Naïve Bayes; RF: random forests.

**Table 4:** Machine learning analysis and statistical comparison through chi square test for proportions after SMOTE implementation.

		Accuracy (%)	Error (%)	Recall (%)	Specificity (%)
Tree	C-SPECT	88.1	11.9	86.2	90.1
	CZT-SPECT	88.1	11.9	86.9	89.3
	*p* value	1.000		0.760	0.731
KNN	C-SPECT	91.9	8.1	83.9	99.8
	CZT-SPECT	91.6	8.4	84.7	98.5
	*p* value	0.858		0.774	0.058
SVM	C-SPECT	91,5	8.5	87,6	95.0
	CZT-SPECT	94.5	5.5	92.2	96.8
	*p* value	**0.016**		**0.028**	0.279
NB	C-SPECT	59.3	40.7	86.7	32.0
	CZT-SPECT	59.0	41.0	87.6	30.3
	*p* value	0.880		0.677	0.599
RF	C-SPECT	93.4	6.6	90.3	94.4
	CZT-SPECT	93.0	7.0	91.0	94.9
	*p* value	0.637		0.720	0.757

Abbreviations. KNN: *K* nearest neighbor; SVM: support vector machine; NB: Naïve Bayes; RF: random forests.

## Data Availability

The dataset used to support the findings of this study have not been made available because of the privacy policy.
